The article "Diagnosis of Chronic Kidney Disease Using Effective Classification Algorithms and Recursive Feature Elimination Techniques" was published in 2021. Journal: J Healthc Eng.

# Diagnosis of Chronic Kidney Disease Using Effective Classification Algorithms and Recursive Feature Elimination Techniques

**DOI:** 10.1155/2021/1004767

**Published:** 2021-06-09

**Authors:** Ebrahime Mohammed Senan, Mosleh Hmoud Al-Adhaileh, Fawaz Waselallah Alsaade, Theyazn H. H. Aldhyani, Ahmed Abdullah Alqarni, Nizar Alsharif, M. Irfan Uddin, Ahmed H. Alahmadi, Mukti E Jadhav, Mohammed Y. Alzahrani

**Affiliations:** ^1^Department of Computer Science and Information Technology, Dr. Babasaheb Ambedkar Marathwada University, Aurangabad, India; ^2^Deanship of E-learning and Distance Education, Hofuf, King Faial University Saudi Arabia, Hofuf, Saudi Arabia; ^3^College of Computer Sciences and Information Technology, King Faisal University, Hofuf, Saudi Arabia; ^4^Community College of Abqaiq, King Faisal University, P.O. Box 400, Hofuf, Al-Ahsa 31982, Saudi Arabia; ^5^Department of Computer Sciences and Information Technology, Albaha University, Al Bahah, Saudi Arabia; ^6^Department of Computer Engineering and Science, Albaha University, Al Bahah, Saudi Arabia; ^7^Institute of Computing, Kohat University of Science and Technology, Kohat, Pakistan; ^8^Department of Computer Science and Information, Taibah University, Medina, Saudi Arabia; ^9^Shri Shivaji Science and Arts College, Chikhli District, Buldana, India

## Abstract

Chronic kidney disease (CKD) is among the top 20 causes of death worldwide and affects approximately 10% of the world adult population. CKD is a disorder that disrupts normal kidney function. Due to the increasing number of people with CKD, effective prediction measures for the early diagnosis of CKD are required. The novelty of this study lies in developing the diagnosis system to detect chronic kidney diseases. This study assists experts in exploring preventive measures for CKD through early diagnosis using machine learning techniques. This study focused on evaluating a dataset collected from 400 patients containing 24 features. The mean and mode statistical analysis methods were used to replace the missing numerical and the nominal values. To choose the most important features, Recursive Feature Elimination (RFE) was applied. Four classification algorithms applied in this study were support vector machine (SVM), *k*-nearest neighbors (KNN), decision tree, and random forest. All the classification algorithms achieved promising performance. The random forest algorithm outperformed all other applied algorithms, reaching an accuracy, precision, recall, and F1-score of 100% for all measures. CKD is a serious life-threatening disease, with high rates of morbidity and mortality. Therefore, artificial intelligence techniques are of great importance in the early detection of CKD. These techniques are supportive of experts and doctors in early diagnosis to avoid developing kidney failure.

## 1. Introduction

Chronic kidney disease (CKD) has received much attention due to its high mortality rate. Chronic diseases have become a concern threatening developing countries, according to the World Health Organization (WHO) [1]. CKD is a kidney disorder treatable in its early stages, but it causes kidney failure in its late stages. In 2016, chronic kidney disease caused the death of 753 million people worldwide, where the number of males died was 336 million, while the number of females died was 417 million [2]. It is called “chronic” disease because the kidney disease begins gradually and lasts for a long time, which affects the functioning of the urinary system. The accumulation of waste products in the blood leads to the emergence of other health problems, which are associated with several symptoms such as high and low blood pressure, diabetes, nerve damage, and bone problems, which lead to cardiovascular disease. Risk factors for CKD patients include diabetes, blood pressure, and cardiovascular disease (CVD) [3]. CKD patients suffer from side effects, especially in the late stages, which damage the nervous and immune system. In developing countries, patients may reach the late stages, so they must undergo dialysis or kidney transplantation. Medical experts determine kidney disease through glomerular filtration rate (GFR), which describes kidney function. GFR is based on information such as age, blood test, gender, and other factors suffered by the patient [4]. Regarding the GFR value, doctors can classify CKD into five stages.  Table 1 shows the different stages of kidney disease development with GFR levels.

Early diagnosis and treatment of chronic kidney disease will prevent its progression to kidney failure. The best way to treat chronic kidney disease is to diagnose it in the early stages, but discovering it in its late stages will lead to kidney failure, which requires continuous dialysis or kidney transplantation to maintain a normal life. In the medical diagnosis of chronic kidney disease, two medical tests are used to detect CKD, which are by a blood test to check the glomerular filtrate or by a urine test to check albumin. Due to the increasing number of chronic kidney patients, the scarcity of specialist physicians, and the high costs of diagnosis and treatment, especially in developing countries, there is a need for computer-assisted diagnostics to help physicians and radiologists in supporting their diagnostic decisions. Artificial intelligence techniques have played a role in the health sector and medical image processing, where machine learning and deep learning techniques have been applied in the processes of disease prediction and disease diagnosis in the early stages. Artificial intelligence (ANN) approaches have played a basic role in the early diagnosis of CKD. Machine learning algorithms are used for the early diagnosis of CKD. The ANN and SVM algorithms are among the most widely used technologies. These technologies have great advantages in diagnosing several fields, including medical diagnosis. The ANN algorithm works like human neurons, which can learn how to operate once properly trained, and its ability to generalize and solve future problems (test data) [5]. However, SVM algorithm depends on experience and examples to assign labels to the class. SVM algorithm basically separates the data by a line that achieves the maximum distance between the class data [6]. Many factors affect kidney performance, which induce CKD, like diabetes, blood pressure, heart disease, some kind of food, and family history.  Figure 1 presents some factors affecting chronic kidney disease.

Pujari et al. [7] presented a system for detecting the stages of CKD through ultrasonography (USG) images. The algorithm works to identify fibrotic cases during different periods. Ahmed et al. [8] proposed a fuzzy expert system to determine whether the urinary system is good or bad. Khamparia et al. [9] studied a stacked autoencoder model to extract the characteristics of CKD and used Softmax to classify the final class. Kim et al. [10] proposed a genetic algorithm (GA) based on neural networks in which the weight vectors were optimized by GA to train NN. The system surpasses traditional neural networks for CKD diagnosis. Vasquez-Morales et al. [11] presented a model based on neural networks to predict whether a person is at risk of developing CKD. Almansour et al. [12] diagnosed a CKD dataset using ANN and SVM algorithms. ANN and SVM reached an accuracy of 99.75% and 97.75%, respectively. Rady and Anwar [13] applied probabilistic neural networks (PNN), multilayer perceptron (MLP), SVM, and radial basis function (RBF) algorithms to diagnose CKD dataset. The PNN algorithm outperformed the MLP, SVM, and RBF algorithms. Kunwar et al. [14] applied two algorithms—naive Bayes and artificial neural networks (ANN)—to diagnose a UCI dataset for CKD. Naive Bayes algorithm outperformed ANN. The accuracy of the naive Bayes algorithm was 100%, while the ANN accuracy was 72.73%. Wibawa et al. [15] applied correlation-based feature selection (CFS) for feature selection, and AdaBoost for ensemble learning was applied to improve CKD diagnosis. The KNN, naive Bayes, and SVM algorithms were applied for CKD dataset diagnosis. Their system achieved the best accuracy when implementing a hybrid between KNN with CFS and AdaBoost by 98.1%. Avci et al. [16] used WEKA software to diagnose the UCI dataset for CKD. The dataset was evaluated using NB, K-Star, SVM, and J48 classifiers. The J48 algorithm outperformed the rest of the algorithms with an accuracy of 99%. Chiu et al. [17] built intelligence models using neural network algorithms to classify CKD. The models included a back-propagation network (BPN), generalized feed forward neural networks (GRNN), and modular neural network (MNN) for the early detection of CKD. The authors proposed hybrid models between the GA and the three mentioned models. Shrivas et al. [18] applied the Union Based Feature Selection Technique (UBFST) to choose the most important features. The selected features were diagnosed by several techniques of machine learning. The aim of the study was to reduce diagnostic time and obtain high diagnostic accuracy. Kunwar et al. [14] used Artificial Neural Network (ANN) and Naive Bayes to evaluate a UCI dataset of 400 patients. The experiment was implemented with RapidMiner tool. Naive Bayes reached a diagnostic accuracy of 100% better than ANN, which reached a diagnostic accuracy of 72.73%. Elhoseny et al. [19] presented a system for healthcare to diagnose CKD through Density Based Feature Selection (DFS) and also a method of Ant Colony Optimization. DFS removes unrelated features that have weak association with the target feature. Abdelaziz et al. [20] presented healthcare service (HCS) system, applying Parallel Particle Swarm Optimization (PPSO), to optimize selection of Virtual Machines (VMs). Then, a new model with linear regression (LR) and neural network (NN) was applied to evaluate the performance of their VMs for diagnosing CKD. Xiong et al. [21] proposed the Las Vegas Wrapper Feature Selection method (LVW-FS) to extract the most important vital features. Ravizza et al. [22] applied a model to test diabetes related to chronic kidney disease. To reduce the dimensions of high data, the Chi-Square statistical method was applied. The model predicts the state of the kidney through some features such as glucose, age, rate of albumin, etc. Sara et al. [23] applied two methods, namely, Hybrid Wrapper and Filter-Based FS (HWFFS) and Feature Selection (FS), to reduce the dimensions of the dataset and select the features associated with CKD strongly. The features extracted from the two methods were then combined, and the hybrid features were classified by using SVM classifier.

The contribution of the current study lies in using Recursive Feature Elimination (RFE) technique with machine learning algorithms to develop system for detecting chronic kidney diseases. The contributions of this paper are summarized as follows:

- We used integrated model to select the most significant representative features by using the Recursive Feature Elimination (RFE) algorithm
- Four machine learning algorithms, namely, SVM, KNN, Decision Tree, and Random Forest, were used to diagnose CKD with promising accuracy
- Highly efficient machine learning techniques for the diagnosis of chronic kidney disease can be popularized with the help of expert physicians

## 2. Materials and Methods

A series of experiments were conducted using machine learning algorithms: SVM, KNN, decision tree, and random forest to evaluate CKD dataset.  Figure 2 shows the general structure of CKD diagnosis in this paper. In preprocessing, the mean method was used to compute the missing numerical values, and the mode method was used to compute the missing nominal values. The features of importance associated with the features of importance for CKD diagnosis were selected using the RFE algorithm. These selected features were fed into classifiers for disease diagnosis. In this study, four classifiers were applied to diagnose CKD: SVM, KNN, decision tree, and random forest. All classifiers showed promising results for diagnosing a dataset into CKD or a normal kidney.

### 2.1. Dataset

The CKD dataset was collected from 400 patients from the University of California, Irvine Machine Learning Repository [24]. The dataset comprises 24 features divided into 11 numeric features and 13 categorical features, in addition to the class features, such as “ckd” and “notckd” for classification. Features include age, blood pressure, specific gravity, albumin, sugar, red blood cells, pus cell, pus cell clumps, bacteria, blood glucose random, blood urea, serum creatinine, sodium, potassium, hemoglobin, packed cell volume, white blood cell count, red blood cell count, hypertension, diabetes mellitus, coronary artery disease, appetite, pedal edema, and anemia. The diagnostic class contains two values: ckd and notckd. All features contained missing values except for the diagnostic feature. The dataset is unbalanced because it contains 250 cases of “ckd” class by 62.5% and 150 cases of “notckd” by 37.5%.

### 2.2. Preprocessing

The dataset contained outliers and noise, so it must be cleaned up in a preprocessing stage. The preprocessing stage included estimating missing values and eliminating noise, such as outliers, normalization, and checking of unbalanced data. Some measurements may be missed when patients are undergoing tests, thereby causing missing values. The dataset contained 158 completed instances, and the remaining instances had missing values. The simplest method to handle missing values is to ignore the record, but it is inappropriate with small dataset. We can use algorithms to compute missing values instead of removing records. The missing values for numerical features can be computed through one of the statistical measures, such as mean, median, and standard deviation. However, the missing values of nominal features can be computed using the mode method, in which the missing value is replaced by the most common value of the features. In this study, the missing numerical features were replaced by the mean method, and a mode method was applied to replace the missing nominal features.  Table 2 shows the statistical analysis of the dataset, such as mean and standard deviation; max and min were introduced for the numerical features in the dataset.  Table 3 shows statistical analysis of numerical feature. While numerical features are the values that can be measured and have two types, either separate or continuous.

### 2.3. Features Selection

After computing the missing values, identifying the important features having a strong and positive correlation with features of importance for disease diagnosis is required. Extracting the vector features eliminates useless features for prediction and those that are irrelevant, which prevents the construction of a robust diagnostic model [25]. In this study, we used the RFE method to extract the most important features of a prediction. The Recursive Feature Elimination (RFE) algorithm is very popular due to its ease of use and configurations and its effectiveness in selecting features in training datasets relevant to predicting target variables and eliminating weak features. The RFE method is used to select the most significant features by finding high correlation between specific features and target (labels).  Table 4 shows the most significant features according to RFE; it is noted that albumin feature has highest correction (17.99%), featured by 14.34%, then the packed cell volume feature by 12.91%, and the serum creatinine feature by 12.09%. RFECV plots the number of features in the dataset along with a cross-validated score and visualizes the selected features is presented in Figure 3.

### 2.4. Classification

Data mining techniques have been used to define new and understandable patterns to construct classification templates [26]. Supervised and unsupervised learning techniques require the construction of models based on prior analysis and are used in medical and clinical diagnostics for classification and regression [27]. Four popular machine learning algorithms used are SVM, KNN, decision tree, and random forest, which give the best diagnostic results. Machine learning techniques work to build predictive/classification models through two stages: the training phase, in which a model is constructed from a set of training data with the expected outputs, and the validation stage, which estimates the quality of the trained models from the validation dataset without the expected output. All algorithms are supervised algorithms that are used to solve classification and regression problems.

#### 2.4.1. Support Vector Machine Classifier

The SVM algorithm primarily creates a line to separate the dataset into classes, enabling it to decide the test data into which classes it belongs. The line or decision boundary is called a hyperplane. The algorithm works on two types: linear and nonlinear. Linear SVM is used when the dataset comprises two classes and is separable. When the dataset is inseparable, a nonlinear SVM is applied, where the algorithm converts the original coordinate area into a separable space. There can be multiple hyperplanes, and the best hyperplane is chosen with the max margin between data points. The dataset closest to the hyperplane is called a support vector.

(1) $$\begin{array}{c} K\left(X,X^{\prime }\right)=\exp\left(-\frac{{\left\|X-X^{\prime }\right\|}^{2}}{2\sigma^{2}}\right), \end{array}$$

where *X*, *X*′ are input data and ‖*X* − *X*′‖^2^ indicates the between the between the input features. *σ* is a free parameter. The Radial Basis Function (RBF) was employed for classification data.

#### 2.4.2. *k*-Nearest Neighbour Classifier

The KNN algorithm works on the similarity between new and stored data points (training points) and classifies the new test point into the most similar class among the available classes. The KNN algorithm is nonparametric, and it is called the lazy learning algorithm, meaning that it does not learn from the training dataset, but rather stores the training dataset. When classifying the new dataset (test data), it classifies the new data based on the value of *k*, where it uses the Euclidean distance to measure the distance between the new point and the stored training points. The new point is classified into a class with the maximum number of neighbors. The Euclidean distance function (Di) was applied to find the nearest neighbored in features vector.

(2) $$\begin{array}{c} D_{i}=\sqrt{\left(x_{1}-x_{2}\right)+{\left(y_{1}-y_{2}\right)}^{2}}, \end{array}$$

where *x*_1_, *x*_2_, *y*_1_, and *y*_2_ are variables for input data.

#### 2.4.3. Decision Tree Classifier

A decision tree algorithm is based on a tree structure. The root node represents the entire dataset, the internal nodes represent the features, the branches represent the decision rules, and the leaf node represents the outcome. A decision tree contains two types of nodes: a decision node, having additional branches, and a leaf node, lacking additional branches. Decisions are performed following the given features. The decision tree compares the feature in the root node with the features' record (real dataset), and based on the comparison, the algorithm takes the decision and moves to the next node. The algorithm compares the features in the second node with the features in the subnodes, and the process continues until it reaches the leaf node.

#### 2.4.4. Random Forest Classifier

The random forest algorithm works according to the principle of ensemble learning by combining several classifiers to improve model performance and solve a complex problem. By the name of the algorithm, it is a classifier that contains some decision trees on subsets of the dataset, and an average is taken to improve the prediction. Instead of relying on a single decision tree for the prediction process, the random forest algorithm takes predictions from each decision tree and relies on the majority vote to make the decision to predict the final outcome. The more tree numbers, the higher the accuracy, and this prevents the overfitting problem. Since the algorithm contains some decision trees to predict the class of a dataset, some trees may predict the correct output while others may not. Therefore, there are two assumptions for the high accuracy of a prediction. First, the feature variable must contain actual values for the algorithm to predict accurate results instead of guessing. Second, the correlation between the predictions of each tree should be very low. Therefore, there are two assumptions for a high accuracy of a prediction. First, the feature variable must contain actual values so that the algorithm can predict accurate results instead of guessing. Second, the correlation between the predictions of each tree should be very low.

Pseudocode of Random forest tree is as follows:

- Find the number of trees for generating, e.g., *K*.
- When *k* (1 < *k* < *K*):
- Feature vector Θ_*K*_ is generated, Θ_*K*_ represents input data generated from creating tree samples
- At this step, construct tree - *h*(*x*, Θ_*K*_)
- Employing any Decision Tree Algorithm
- At this step, each tree casts 1 vote for class *y*
- The class *y* is classified by choosing the class with maximum votes

## 3. Experiment Environment Setup

This section presents the results of the developing system.

### 3.1. Environment Setup

The system has been developed by using different environments.  Table 5 shows the environment setup of the developing system.

### 3.2. Evaluation Metrics

Evaluation metrics were used to evaluate the performance of the four classifiers. One of these measures is through the confusion matrix, from which the accuracy, precision, recall, and F1-score are extracted by computing the correctly classified samples (TP and TN) and the incorrectly classified samples (FP and FN), as shown in the following equations [28]:

(3) $$\begin{array}{c} \text{accuracy}=\frac{\text{TN}+\text{TP}}{\text{TN}+\text{TP}+\text{FN}+\text{FP}}*100\%, \end{array}$$

(4) $$\begin{array}{c} \text{precision}=\frac{\text{TP}}{\text{TP}+\text{FP}}*100\%, \end{array}$$

(5) $$\begin{array}{c} \text{recall}=\frac{\text{TP}}{\text{TP}+\text{FN}}*100\%, \end{array}$$

(6) $$\begin{array}{c} F1-\text{score}=2*\frac{\text{precision}*\text{recall}}{\text{precision}*\text{recall}}*100, \end{array}$$

where TN is True Negative, TP is True Positive, FN is False Negative, and FP is False Positive.

### 3.3. Splitting Dataset

The dataset was divided into 75% for training and 25 for testing and validation.  Table 6 shows the splitting data.

## 4. Results

The random forest algorithm classified all positive and negative samples correctly, as positive samples were correctly classified 250 samples (TP), and all negative samples (TN) were classified for 150 samples correctly. While the SVM, KNN, and Decision Tree algorithms rated the positive (TP) samples by 94.74%, 97.37%, and 98.68%, respectively, that is, with an error (TN) 5.26%, 2.63%, and 1.32%, respectively.  Table 6 shows the results obtained from the four classifiers. The random forest algorithm outperformed the rest of the classifiers, reaching an accuracy, precision, recall, and F1-score of 100% for all measures. It was followed by the decision tree algorithm, which reached the accuracy, precision, recall, and F1-score with a score of 99.17%, 100%, 98.68%, and 99.34%, respectively. Then, the KNN algorithm came up with accuracy, precision, recall, and F1-score of 98.33%, 100% 97.37%, and 98.67%, respectively. Finally, the SVM accuracy, precision, recall, and F1-score algorithm scored 96.67%, 92%, 94.74%, and 97.30%, respectively.

The performance of the proposed systems was evaluated through several previous related studies, as shown in Table 7. It is noted that the existing studies have obtained the lowest accuracy; the accuracy ranges of existing studies are between 96.8% and 66.3%, while the proposed system has obtained accuracy of 100% with random forest tree method. Finally, it is observed that the proposed has optimal results compared with existing systems.

Twenty-four numerical and nominal features were introduced from 400 patients with CKD. Due to the neglect of some tests for some patients, some computation methods were applied to solve this problem. To solve the missing numerical values, mean method was used; for missing nominal values, the mode method was used. As Figure 4 shows a correlation between different features, the figure shows positive and negative correlation. There is a positive correlation, for example, between specific gravity with red blood cell count, packed cell volume, and hemoglobin; between sugar with blood glucose random; between blood urea and serum creatinine; and between hemoglobin with red blood cell count and packed cell volume. There is also a negative correlation, for example, between albumin and blood urea with red blood cell count, packed cell volume, and hemoglobin and between serum creatinine and sodium.

### 4.1. Results and Discussion

The dataset is randomly divided into 75% for training and 25% for testing and validation. The Recursive Feature Elimination method was presented to select the irrelevant subset features. Then, the select features were processed by employing classifiers for diagnosis of CKD. A comparative analysis between the proposed system and existing approaches is presented in Table 8. It is noted that the proposed system has achieved promising results. We have used RFE algorithm for finding the best relationships between each feature with the target features and works to prioritize the features and give each feature a percentage based on the correlation with the target feature.  Figure 5 displays the performance of the proposed system against existing systems, where the accuracy in the existing systems reached a ratio between 95.84% and 66.3%, while the accuracy of our systems reached between 100% by random forest and 97.3% by SVM.

## 5. Conclusion

This study provided insight into the diagnosis of CKD patients to tackle their condition and receive treatment in the early stages of the disease. The dataset was collected from 400 patients containing 24 features. The dataset was divided into 75% training and 25% testing and validation. The dataset was processed to remove outliers and replace missing numerical and nominal values using mean and mode statistical measures, respectively. The RFE algorithm was applied to select the most strongly representative features of CKD. Selected features were fed into classification algorithms: SVM, KNN, decision tree, and random forest. The parameters of all classifiers were tuned to perform the best classification, so all algorithms reached promising results. The random forest algorithm outperformed all other algorithms, achieving an accuracy, precision, recall, and F1-score of 100% for all measures. The system was examined and evaluated through multiclass statistical analysis, and the empirical results of SVM, KNN, and decision tree algorithms found significant values of 96.67%, 98.33%, and 99.17% with respect to accuracy metric.

## Figures and Tables

**Figure 1:** Factors affecting chronic kidney disease.

**Figure 2:** The proposed system for the diagnosis of CKD.

**Figure 3:** Number of features vs. cross-validated score.

**Figure 4:** Correlation between different features.

**Figure 5:** Comparison of system's performance on diagnostic accuracy in the two datasets.

**Table 1:** The stages of development of CKD.

Stage	Description	Glomerular filtration rate (GFR) (mL/min/1.73 m^2^)	Treatment stage
1	Kidney function is normal	≥90	Observation, blood pressure control
2	Kidney damage is mild	60–89	Observation, blood pressure control and risk factors
3	Kidney damage is moderate	30–59	Observation, blood pressure control and risk factors
4	Kidney damage is severe	15–29	Planning for end-stage renal failure
5	Established kidney failure	≤ 15	Treatment choices

**Table 2:** Statistical analysis of the dataset of numerical features.

Features	Mean	Standard deviation	Max	Min
Age	51.483	17.21	90	2
Blood glucose random	148.037	76.583	490	22
Serum creatinine	3.072	4.512	76	0.4
Blood pressure	76.469	13.756	180	50
Blood urea	57.426	49.987	391	1.5
Potassium	4.627	2.92	47	2.5
Packed cell volume	38.884	8.762	54	9
Sodium	137.529	9.908	163	4.5
Hemoglobin	12.526	2.815	17.8	3.1
White blood cell count	8406.12	2823.35	26400	2200
Red blood cell count	4.707	0.89	8	2.1

**Table 3:** Statistical analysis of the dataset of nominal features.

Features	Label	Count
Albumin	0	245
	1	44
	2	43
	3	43
	4	24
	5	1

Specific gravity	1.005	7
	1.01	84
	1.015	75
	1.02	153
	1.025	81

Sugar	0	339
	1	13
	2	18
	3	14
	4	13
	5	3

Pus cell	Normal	324
	Abnormal	76

Red blood cells	Normal	353
	Abnormal	47

Bacteria	Present	22
	Not present	378

Pus cell clumps	Present	42
	Not present	358

Diabetes mellitus	Yes	137
	No	263

Hypertension	Yes	147
	No	253

Edema	Yes	76
	No	324

Coronary artery disease	Yes	34
	No	366

Anemia	Yes	60
	No	340

Appetite	Good	318
	Poor	82

**Table 4:** The importance of predictive variables in diagnosing CKD.

Features	Priority ratio (%)
al	17.99
hemo	14.34
pcv	12.91
sc	12.09
rc	7.51
bu	6.56
sg	6.08
pcv	5.60
htn	4.64
bgr	3.48
dm	3.20
pe	1.25
wc	1.01
sod	0.92
rbc	0.91
bp	0.39
su	0.35
appet	0.28
ba	0.18
age	0.18
cad	0.09
pcc	0.06
pot	0.00
ane	0.00

**Table 5:** Environment setup of the proposed system.

Resource	Details
CPU	Core i5 Gen6
RAM	8 GB
GPU	4 GB
Software	Python

**Table 6:** Splitting dataset.

Dataset	Numbers
Training	300 patients
Testing and validation	100 patients

**Table 7:** Results of diagnosing CKD using four machine learning algorithms.

Classifiers	SVM	KNN	Decision tree	Random forest
Accuracy %	96.67	98.33	99.17	100.00
Precision %	92.00	100.00	100.00	100.00
Recall %	94.74	97.37	98.68	100.00
F1-score%	97.30	98.67	99.34	100.00

**Table 8:** Comparison of the performance of our proposed system with previous studies.

Previous studies	Accuracy %	Precision %	Recall %	F1-score %
Hore et al. [29]	92.54	85.71	96	90.56
Vasquez-Morales et al. [11]	92	93	90	91
Rady and Anwar [13]	95.84	84.06	93.55	88.55
Elhoseny et al. [19]	85		88	88
Ogunleye and Wang [30]	96.8		87	93
Khan et al. [31]	95.75	96.2	95.8	95.8
Chittora et al. [32]	90.73	83.34	93	88.05
Jongbo et al. [33]	89.2	97.72	97.8	
Harimoorthy and Thangavelu [34]	66.3	65.9	65.9	
Proposed model (random forest)	100	100	100	100
Proposed model (decision tree)	99.34	98.68	100	99.17
Proposed model (KNN)	98.33	100	97.37	98.67
Proposed model (SVM)	97.3	94.74	92	96.67

## Data Availability

Data were collected from UCI Machine Learning Repository, School of Information and Computer Science, University of California, Irvine, CA, USA (http://archive.ics.uci.edu/ml).
